The article "Flow Simulation in the Upper Respiratory Tract of Two Obstructive Sleep Apnea Patients with Successful and Failed Surgery" was published in 2021. Journal: Comput Math Methods Med.

# Flow Simulation in the Upper Respiratory Tract of Two Obstructive Sleep Apnea Patients with Successful and Failed Surgery

**DOI:** 10.1155/2021/6683828

**Published:** 2021-05-07

**Authors:** Jiacun Shao, Weiwei Yan, Yang Liu, Mingzhen Lu

**Affiliations:** ^1^College of Metrology and Measurement Engineering, China Jiliang University, Hangzhou, China; ^2^Department of Mechanical Engineering, The Hong Kong Polytechnic University, Kowloon, Hong Kong

## Abstract

Obstructive sleep apnea (OSA) is a common disorder which may need to be treated by the upper respiratory tract (URT) surgery. To increase the success rate of the URT surgery, it is crucial to understand the flow features in the URT models. In this work, the turbulent flow characteristics in four 3D anatomically accurate URT models reconstructed from two OSA subjects with successful and failed surgery are numerically studied by the large-eddy simulation (LES) and unsteady Reynolds-averaged Navier-Stokes (RANS). The features of velocity fields, pressure fields, and wall shear stress fields as well as the spectral analysis of wall shear stress between successful and failed surgery are explored. The results indicate that LES is capable of capturing flow patterns and flow oscillation and is effective for OSA surgery prediction. Even if the unsteady RANS can obtain the correct pressure drop across the airways, it may not be appropriate to be used for surgery prediction. Moreover, it is found that the quality of oscillating signal of wall shear stress is a key factor in surgery prediction. In a successful surgery, the wall shear stress oscillation is always strong, and the oscillating signal can perform a dominant frequency near 3~5 Hz, while in a failed surgery it does not show this clear intrinsic property. The results not only will gain new insights in the URT surgical planning but also will improve the prediction of surgical outcome for OSA patients.

## 1. Introduction

Obstructive sleep apnea (OSA) is a disease characterized by repetitive episodes of the upper respiratory tract (URT) obstruction during sleep, which is related to a multitude of adverse health conditions [1, 2]. It is a causative factor for the development of systemic hypertension, cardiac dysrhythmias, stroke, angina, and diabetes, to name a few [3, 4]. The surgery, aimed at improving the size or tone of the URT, is regarded as the first choice of OSA treatment. The main idea of the URT surgery is to eliminate the area of obstruction by dismissing the uvula and some of the peripheral soft palate. However, the success rate of the surgery is always not satisfactory, about 50% only. The postoperative complications are often a dilemma during the operation of how much tissue to remove: too little is ineffective, too much makes OSA worse [5]. Accurate prediction of tissue resection for OSA treatment is urgently needed. Appropriate surgical planning should be based on the understanding of pathophysiology of URT obstruction. Due to the complexity of realistic OSA URT, it is expensive and difficult to study airway flow experimentally, no matter in vivo or in vitro. In contrast, computational fluid dynamics (CFD) has become a powerful tool for analyzing airway flow patterns and obtaining quantitative and qualitative information about flow variables [6–8], which will help to comprehend the pathophysiology of URT obstruction, to plan surgical strategies for OSA diseases, and to predict surgical outcome of OSA patients.

The article "Flow Simulation in the Upper Respiratory Tract of Two Obstructive Sleep Apnea Patients with Successful and Failed Surgery" was published in 2021. Journal: Comput Math Methods Med.

Although extensive numerical studies on flow patterns in the human airways have been conducted [8–11], few researchers have explored the URT flow of OSA patients using the CFD [12–15]. Since the morphology of realistic OSA URT is very complex, the flow in it is expected to be turbulent [16]. There are three common techniques to model turbulent airway flow, i.e., direct numerical simulation (DNS), Reynolds-averaged Navier-Stokes (RANS), and large-eddy simulation (LES). Wang and Elghobashi executed a DNS research on flow characteristics in two patient-specific URTs. They revealed that the amplitude and frequency of pressure fluctuations were reduced in the obstructed location [12]. Although the DNS is the most accurate technique for turbulent flow modeling, it is rather expensive to simulate turbulent airway flow at high Reynolds number. A numerical study on flow patterns and aerodynamic force in the URT of an OSA patient was also performed via the RANS [13]. It was observed that the turbulent jet generated at the velopharynx due to regional restriction was the most striking feature in the OSA pharyngeal airway. Recently, our group portrayed the transitional and turbulent airway flow patterns in an obstructed OSA URT model utilizing the LES [15]. It was concluded that the LES was capable of providing information for understanding the pathogenesis of OSA syndrome.

There exist different views on the RANS and LES for flow simulation in the human airways. In the previous studies, most CFD analyses were based on the RANS solvers using two-equation turbulence models [13, 17–20]. Backer et al. indicated that the low Reynolds number (LRN) k-*ω* model could accurately predict pressure drops and velocity profiles in the URT models [17]. Mihaescu et al. compared the LES and steady RANS (including k-*ε* and k-*ω* models) in flow simulation in a realistic pharyngeal airway, but made a contrary conclusion [18]. They reported that the steady RANS might not be the proper tool to study flows in the URTs, but the LES could provide an increased level of detail and accuracy for the unsteady, separated, or vortical turbulent flow situations. Bass and Longest analyzed the effects of different turbulent models (including LRN k-*ω* and LES models) on microparticle deposition features in the URTs [19]. They stated that the more computationally efficient LRN k-*ω* was capable of providing deposition results that were comparable to the LES. In view of the above arguments, we numerically study the flow features in four realistic URT models reconstructed from two OSA subjects both before and after surgery by adopting the LES and three unsteady RANS turbulent models (including unsteady standard k-*ε*, standard k-*ω*, and k-*ω* SST). In our previous work, we found that there existed flow oscillation induced by flow separation at the larynx which played an important role in activating the mechanoreceptors which was crucial for OSA subjects [21]. Thus, in this work, we also numerically explore the flow oscillation characteristics in the URT models of two OSA subjects with successful and failed surgery. We expect to gain new insights in the URT surgical planning and have the potential for improving the predicting of OSA surgical outcome.

The article "Flow Simulation in the Upper Respiratory Tract of Two Obstructive Sleep Apnea Patients with Successful and Failed Surgery" was published in 2021. Journal: Comput Math Methods Med.

## 2. Methods

### 2.1. Construction of URT Models

The major structure of human URT can be seen in Figure 1. In this study, two adult males (subject 1: 38 years old, BMI 25.7, 76 kg; subject 2: 45 years old, BMI 26.4, 80 kg) who suffered severe OSA disease before treatment and had the uvulopalatopharyngoplasty surgery which removed or reduced parts of the soft palate and uvula are selected. The thoracic CT scan just needs a few seconds and is fast enough for patients to hold their breath; thus, it is used for presurgery at first and for postsurgery six months after surgery. The CT scan images are obtained in the axial plane with a resolution of 0.7 × 0.7 mm^2^ and a slice thickness of 0.625 mm. Based on the CT scan images of two OSA subjects, 3D point cloud data of URT models are reconstructed via the image processing software Mimics 17.0.  Figure 2 exhibits the side view and front view of four 3D anatomically accurate URT models, where (a1, a2) and (b1, b2) denote the models of subject 1 before and after surgery and (c1, c2) and (d1, d2) indicate the models of subject 2 before and after surgery.

The severity of OSA disease is defined by the apnea-hyponea index (AHI), suggesting the number of apneas and hypopneas per hour. The severity indices of OSA syndrome are tabulated in Table 1 [22], and Table 2 shows the AHI measurement, minimal cross-sectional area near the retropalate, maximal cross-sectional area in the oropharynx, and area ratio (min area/max area) of two OSA subjects before and after surgery. For subject 1, the minimal cross-sectional area is expanded from 53 mm^2^ to 100 mm^2^, as twice as before treatment. Meanwhile, AHI reduces from 64.8 (severe OSA) to 15.8 (mild OSA), revealing an acceptable surgery outcome. For subject 2, the minimal cross-sectional area is enlarged from 46 mm^2^ to 318 mm^2^, increased by five times. However, the reduction of AHI from 60.7 (severe OSA) to 23.9 (moderate OSA) shows an unsatisfactory surgery outcome that the sleep hypopnea problem of the patient could not disappear completely. A strong correlation between AHI and the area ratio of minimal cross-section near the retropalate and maximal cross-section behind the tongue base can be found. However, it is worthy to note that there are no correlations between AHI change and the increase in minimal cross-sectional area, revealing that the overwidened URT may not make the AHI lower and benefit OSA patients.

The article "Flow Simulation in the Upper Respiratory Tract of Two Obstructive Sleep Apnea Patients with Successful and Failed Surgery" was published in 2021. Journal: Comput Math Methods Med.

### 2.2. Numerical Methods

Since the real flow in the URT is transient, the results of the unsteady RANS should be more accurate than the steady RANS, and therefore, we compare the unsteady RANS (including standard k-*ε*, standard k-*ω*, and k-*ω* SST) and LES results in four URT models of two OSA subjects before and after surgery. In the unsteady RANS, the velocity is defined as

(1) $$\begin{array}{c} \bar{U}=\frac{1}{2T}\int_{-T}^{T}U\left(t\right)dt,\;U=\bar{U}+u^{\prime \prime }, \end{array}$$

where the velocity *U* is consisted of the mean component $\bar{U}$ and the fluctuating component *u*^″^. The unsteady RANS equations in incompressible form are [23]

(2) $$\begin{array}{c} \frac{\partial {\bar{U}}_{i}}{\partial x_{i}}=0,\\ \frac{\partial {\bar{U}}_{i}}{\partial t}+{\bar{U}}_{j}\frac{\partial {\bar{U}}_{i}}{\partial x_{j}}=-\frac{1}{\rho }\frac{\partial \bar{P}}{\partial x_{i}}+\nu \frac{\partial^{2}{\bar{U}}_{i}}{\partial x_{j}\partial x_{j}}-\frac{\partial \bar{u_{i}^{\prime \prime }u_{j}^{\prime \prime }}}{\partial x_{j}}, \end{array}$$

where the mean dependent variables in Equation (2) are not only a function of space but also a function of time, namely,

(3) $$\begin{array}{c} {\bar{U}}_{i}={\bar{U}}_{i}\left(x,y,z,t\right),\\ \bar{P}=\bar{P}\left(x,y,x,t\right),\\ \;\bar{u_{i}^{\prime \prime }u_{j}^{\prime \prime }}=\bar{u_{i}^{\prime \prime }u_{j}^{\prime \prime }}\left(x,y,x,t\right). \end{array}$$

We can see the averaged components are still a function of time, and thus, the results from the unsteady RANS are unsteady.

In the LES modeling, the filtering operation $\bar{\varphi }\left(\text{x}\right)$ for a variable *x* is provided by

(4) $$\begin{array}{c} \bar{\varphi }\left(\text{x}\right)=\frac{1}{V}\int_{V}\varphi \left({\text{x}}^{\prime }\right)G\left(\text{x},{\text{x}}^{\prime }\right)d{\text{x}}^{\prime }, \end{array}$$

where *V* is the volume of a computational cell, and the filter function *G*(x, x′) is defined as

(5) $$\begin{array}{c} G\left(x,x^{\prime }\right)=\left\{\begin{array}{cc} 1, & \text{for }x^{\prime }\in V,\\ 0, & \text{otherwise}. \end{array}\right. \end{array}$$

The filtering process effectively filters out the eddies whose scales are smaller than the filter width or grid spacing. The filtered Navier-Stokes equations can be written as

(6) $$\begin{array}{c} \nabla \bar{u}=0,\\ \rho_{\text{f}}\frac{\partial \bar{u}}{\partial t}+\rho \bar{u}\cdot \nabla \bar{u}=-\nabla \bar{p}+\mu_{f}\nabla^{2}\bar{u}, \end{array}$$

where $\bar{u}$ and $\bar{p}$ are the filtered air velocity and pressure, *ρ*_f_ and *μ*_f_ are the air density and viscosity, and *t* is the time. *μ*_*f*_ is the effective viscosity which is unknown and will be modeled by the subgrid scale (SGS) model.

The article "Flow Simulation in the Upper Respiratory Tract of Two Obstructive Sleep Apnea Patients with Successful and Failed Surgery" was published in 2021. Journal: Comput Math Methods Med.

The numerical simulations are carried out by the CFD solver ANSYS-FLUENT 2019. The mesh generator ICEM is utilized to reconstruct airway geometry and to generate meshes. For each URT model, the hybrid hexahedral and tetrahedral computational meshes are used. Compared to the tetrahedral meshes, the hexahedral meshes can evidently reduce the number of meshes and the amount of computation. Thus, in our simulations, the hexahedral meshes are employed inside the URT model domains. Because of the complexity of the structures of four URT models, the tetrahedral meshes are adopted near the wall surfaces to establish good mesh quality there. Besides, the refined meshes are executed in the narrow pharynx and larynx to enhance the solutions in those regions. To accurately capture the flow behavior near the walls, we also conduct mesh refinements near the wall surfaces. *y*+ of the first layer meshes are ensured smaller than 1 according to the requirement of the LES method. Here, *y*+ is a dimensional wall distance defined as

(7) $$\begin{array}{c} y^{+}=\frac{y}{\nu_{f}}\sqrt{\frac{\tau_{w}}{\rho_{f}}}, \end{array}$$

where *y* is the distance to the nearest wall, *ν*_*f*_ is the kinematic viscosity of the air, and *τ*_*w*_ is the wall shear stress.

We attempt to study the inspiratory process with tidal volume 700 ml and the breathing frequency 12 cycles per minute following a sinusoid. The flow is assumed as incompressible flow due to the very low Mach number. The second-order finite-volume schemes are employed to discretize the governing equations (Equation (6)). The time integration is executed using the second-order implicit discretization. The coupling between pressure and velocity fields is performed through the SIMPLE algorithm. In the inlet, the initial velocity is calculated based on the nostril area, and the pressure boundary condition in the outlet is set as zero. The no-slip boundary condition is applied on the surface of the whole airway, and the time step is set to be 0.001 s. The amount of the cell quantity in the computational model is about 3.4 × 10^6^ for subject 1 and 3.7 × 10^6^ for subject 2 both before and after surgery. The computations are achieved using the parallel computing function of a computer. It takes about 12~13 hours to finish a simulation case. The numerical results of velocity in all the URT models are mesh-convergent to within a prescribed tolerance (~0.2%).

The article "Flow Simulation in the Upper Respiratory Tract of Two Obstructive Sleep Apnea Patients with Successful and Failed Surgery" was published in 2021. Journal: Comput Math Methods Med.

### 2.3. Fast Fourier Transformation

The time series after simulation are analyzed by the fast Fourier transformation (FFT). For a real signal *f*(*t*), if we regard it as an ergodic process, its autocorrelation is defined by [24]

(8) $$\begin{array}{c} R\left(\tau \right)=\underset{T\to \infty }{\lim}\frac{1}{T}\int_{-T/2}^{T/2}f\left(t\right)f\left(t-\tau \right)dt, \end{array}$$

and its correlation coefficient is defined by

(9) $$\begin{array}{c} r\left(\tau \right)=\frac{\underset{T\to \infty }{\lim}\left(1/T\right)\int_{-T/2}^{T/2}\left[f\left(t\right)-\mu \right]\left[f\left(t-\tau \right)-\mu \right]dt}{\sigma^{2}}, \end{array}$$

where *μ* and *σ* are the mean and variance of the signal *f*(*t*) and given by

(10) $$\begin{array}{c} \mu =\underset{T\to \infty }{\lim}\frac{1}{T}\int_{-T/2}^{T/2}f\left(t\right)dt,\\ \sigma^{2}=\underset{T\to \infty }{\lim}\frac{1}{T}\int_{-T/2}^{T/2}{\left[f\left(t\right)-\mu \right]}^{2}dt. \end{array}$$

The power spectral density (PSD) can be obtained by imposing Fourier transform (FT) on *R*(*τ*) [25]

(11) $$\begin{array}{c} S\left(\omega \right)=\int_{-\infty }^{\infty }R\left(\tau \right)e^{-i\omega \tau }d\tau . \end{array}$$

On the other hand, if we impose on *r*(*τ*), since *r*(*τ*) = (1/*σ*^2^)*R*(*τ*) − (*μ*^2^/*σ*^2^), we can get

(12) $$\begin{array}{c} s\left(\omega \right)=\int_{-\infty }^{\infty }\left[\frac{1}{\sigma^{2}}R\left(\tau \right)-\frac{\mu^{2}}{\sigma^{2}}\right]e^{-i\omega \tau }d\tau =\frac{1}{\sigma^{2}}S\left(\omega \right)-2\pi \frac{\mu^{2}}{\sigma^{2}}\delta \left(\omega \right), \end{array}$$

where *δ*(*ω*) is the Dirac function. In this study, we also call *s*(*ω*) as the PSD.

## 3. Results and Discussion

### 3.1. Velocity Field Characteristics

Utilizing the LES and three unsteady RANS models, the velocity fields, pressure fields, and wall shear stress fields in four URT models for both pre- and postsurgery are numerically investigated. The axial velocity distribution and axial velocity streamline distribution during inspiration along the sagittal plane for two OSA subjects are illustrated in Figures 3 and 4, respectively. Before surgery, it is found that all the turbulent models can capture a jet-like axial velocity which increases from the minimal cross-sectional area due to the anatomical narrowed airway near the soft palate. The discrepancies are mainly seen in the axial velocity streamlines downstream of the minimal cross-sectional area. Before surgery, the LES is capable of capturing more than two vortexes (Figures 3(d2) and 4(d2)), which are considered as an important factor in the airway occlusion in the anterior side. However, only two vortexes can be observed for the k-*ω* results (Figures 3(b2)–3(c2)) and just one for the k-*ε* results (Figure 3(a2)) for subject 1. For subject 2, all the unsteady RANS models can obtain two large vortexes near the downstream of the minimal cross-sectional area and epiglottis (Figures 4(a2)–4(c2)). Compared to the unsteady RANS results, the LES results exhibit more small random vortexes and a longer axial velocity increasing region along the posterior side of the sagittal plane (Figures 3(d1) and 4(d1)). After surgery, due to the variation of airway morphology, the differences emerged in the anterior side: all the four turbulent models can capture a large vortex downstream of the minimal cross-sectional area for both subjects (Figures 3(e2)–3(h2) and 4(e2)–4(h2)) except for an additional vortex found near the epiglottis in subject 2 (Figure 4(h2)).

The article "Flow Simulation in the Upper Respiratory Tract of Two Obstructive Sleep Apnea Patients with Successful and Failed Surgery" was published in 2021. Journal: Comput Math Methods Med.

Figures 5 and 6 illustrate the axial velocity contour at two cross-sectional planes in the URT models of two OSA subjects before and after treatment. The maximal axial velocity can be observed by all the turbulent models at the minimal cross-sectional area, and the flow patterns seem similar for all the turbulent models for two subjects. For the downstream plane, it is found that the flow patterns obtained by the unsteady RANS, especially for two subjects before surgery, are quite different in the location of the flow separation region from that by the LES (Figures 5(a1)–5(d1) and 6(a1)–6(d1)). However, for the results after surgery, although the k-*ε* results are still different in the flow separation region from the LES results, the flow patterns shaped by the k-*ω* models appear to be close to the LES results (Figures 5(a2)–5(d2) and 6(a2)–6(d2)).

### 3.2. Pressure Field Characteristics

The variations of the mean static pressure distribution corresponding to their cross-sectional area from the nasopharynx to the epiglottis for two OSA subjects are also studied by the LES and unsteady RANS. For subject 1, as shown in Figure 7, the surgery changes the morphology of the airway significantly. The minimal cross-sectional area in the retropalatal region (collapse region for OSA) is widened from nearly 53 mm^2^ to 100 mm^2^, and meanwhile, the narrowest cross-sectional area moves upward after treatment. Before surgery, the static pressure from the nasopharynx to the minimal cross-sectional area decreases dramatically from about 35 Pa to -5 Pa for all the turbulent models. After treatment, due to the expansion of the obstructed structure, the value of the static pressure changes obviously. However, the pressure drop between the above two regions is almost the same; it maintains the value of nearly 7 Pa for all the turbulent models. This indicates that all the turbulent models can capture the pressure drop which is considered as an important factor to evaluate the collapse of URT.

The article "Flow Simulation in the Upper Respiratory Tract of Two Obstructive Sleep Apnea Patients with Successful and Failed Surgery" was published in 2021. Journal: Comput Math Methods Med.

For subject 2, as shown in Figure 8, the minimal cross-sectional area is widened by five times (from 46 mm^2^ to 318 mm^2^) after treatment. Before surgery, the pressure drop in the area from the nasopharynx to the minimal cross-sectional area is quite large due to the large negative pressure induced by the high-speed jet flow, and the pressure drop is more than 60 Pa. After treatment, the pressure drop decreases significantly to less than 0.5 Pa. It can be clearly observed that, even though the pressure value is different with different turbulent models, the pressure profile along the airway is almost the same for all the turbulent models leading to the same pressure drop across the airways.

### 3.3. Shear Stress Field Characteristics

It was reported that the central respiratory pattern generator required an external stimulus to activate respiratory events, and input signals emanate not only from chemoreceptors but also from mechanoreceptors in the human airways [26]. The flow oscillation could trigger the reflex of respiratory muscles. In our previous work, we have found that there exists flow oscillation in the URT which is induced by the flow separation downstream of the minimal cross-sectional area, and the flow oscillation is stronger in the normal subjects, but weak in the abnormal subjects [21]. This oscillating signal may be an external stimulus to the mechanoreceptors or the reflection of the URT dilator muscles. In this study, we also compare the oscillation of wall shear stress based on the LES and unsteady RANS modeling. Figures 9 and 10 display the time history of wall shear stress at one point located at the anterior side of cross section B near the oropharynx for two OSA subjects before and after surgery. It is clearly observed that the LES is capable of capturing the oscillation of wall shear stress quite well, while the unsteady RANS captures very little wall shear stress oscillation. This phenomenon may contribute to the mean component of the velocity in the unsteady RANS in Equation (1).

The article "Flow Simulation in the Upper Respiratory Tract of Two Obstructive Sleep Apnea Patients with Successful and Failed Surgery" was published in 2021. Journal: Comput Math Methods Med.

Since the LES has an advantage over the unsteady RANS in capturing flow oscillation in the human airways, we further conduct the spectral analysis on the wall shear stress time series obtained from the LES modeling.  Figure 11 shows the wall shear stress time series and spectral analysis. The monitoring point is selected at the anterior side of cross section B near the oropharynx. For subject 1 with successful surgery, as exhibited in Figure 11(a), it is observed that the fluctuation of the wall shear stress in that point after surgery is much stronger than that before surgery, which means that the flow oscillation is heightened and the activation to the URT dilator muscles is also strengthened. However, for subject 2 with failed surgery, as shown in Figure 11(b), the wall shear stress fluctuates less after treatment than that before surgery, indicating that the stimulus to the respiratory events is evenly suppressed. Thus, the AHI of subject 2 after surgery is higher than that of subject 1.

In our previous research, we have found from the experiment that the inspiratory flow oscillation can generate a periodic signal with major frequency around 3~5 Hz, an intrinsic property of breathing in the normal subjects [21]. This flow oscillation signal may be the afferent stimulus to the reflex of mechanoreceptors. From the FFT analysis of the wall shear stress, one can find that the present results are consistent with our previous study. As shown in Figure 12(a), the better surgical outcome model performs a dominant frequency near 3 Hz after surgery in subject 1. For subject 2, it can be seen from Figure 12(b) that the PSD after surgery does not show this clear intrinsic property. This can reflect the differences in the surgical outcome as well.

## 4. Conclusion

In this work, the turbulent flow characteristics in four 3D anatomically accurate URT models reconstructed from two OSA subjects with successful and failed surgery are numerically studied. The LES and three unsteady RANS with two-equation turbulence models, including standard k-*ε*, standard k-*ω*, and k-*ω* SST, are adopted to conduct the simulations. Particularly, the features of flow velocity fields, pressure fields, and wall shear stress fields as well as the spectral analysis on the wall shear stress between successful and failed surgery are explored. These results not only will obtain new insights in the surgical planning but also will improve the prediction of the surgical outcome for OSA patients. The simulation results lead to the following conclusions:

1. Before surgery, a strong jet flow is induced and causes several complex recirculation zones downstream of the minimal cross-sectional area. The LES can capture more than two recirculation zones, and the standard k-*ω* and k-*ω* SST can capture two recirculation zones, but only one of these recirculation zones can be captured by the standard k-*ε*. After surgery, the URT models are widened and the jet flow is attenuated. The flow separation induces a main recirculation flow downstream of the minimal cross-sectional area. All the turbulent models can capture this main recirculation zone
2. The pressure drop is an important factor to evaluate the collapse of human airways. For all the four URT models, although the pressure value is different with different turbulent models, the LES and three unsteady RANS models can obtain the same pressure drop across the airways, suggesting that the unsteady RANS has the same capability for the mean pressure simulation compared with the LES
3. The LES can well simulate the oscillation of wall shear stress, while only little wall shear stress fluctuation can be captured by the unsteady RANS. The oscillating wall shear stress can serve as the measurement to quantify the surgical outcome of OSA subjects. In a successful surgery, the wall shear stress oscillation is always strong which denotes intense activation to the URT dilator muscles, and the oscillating signal can perform a dominant frequency near 3~5 Hz. However, in a failed surgery, the wall shear stress fluctuates less which means the stimulus to respiratory events is evenly suppressed, and the oscillating wall shear stress cannot exhibit a major frequency near 3~5 Hz

The article "Flow Simulation in the Upper Respiratory Tract of Two Obstructive Sleep Apnea Patients with Successful and Failed Surgery" was published in 2021. Journal: Comput Math Methods Med.

## Figures and Tables

**Figure 1:** Major structure of URT.

**Figure 2:** Four URT models: (a1, a2) subject 1 before surgery, (b1, b2) subject 1 after surgery, (c1, c2) subject 2 before surgery, and (d1, d2) subject 2 after surgery. Section A is the minimal cross section, and section B is the cross section near the larynx. (a1–d1) Side view; (a2–d2) front view.

**Figure 3:** (a1–h1) Axial velocity distribution and (a2–h2) axial velocity streamline distribution in the sagittal plane for subject 1 (a1–d1, a2–d2) before surgery and (e1–h1, e2–h2) after surgery. (a1, a2, e1, e2) Standard k-*ε* solution; (b1, b2, f1, f2) standard k-*ω* solution; (c1, c2, g1, g2) k-*ω* SST solution; (d1, d2, h1, h2) LES solution.

**Figure 4:** (a1–h1) Axial velocity distribution and (a2–h2) axial velocity streamline distribution in the sagittal plane for subject 2 (a1–d1, a2–d2) before surgery and (e1–h1, e2–h2) after surgery. (a1, a2, e1, e2) Standard k-*ε* solution; (b1, b2, f1, f2) standard k-*ω* solution; (c1, c2, g1, g2) k-*ω* SST solution; (d1, d2, h1, h2) LES solution.

**Figure 5:** Axial velocity distribution (m/s) in the minimum cross-sectional plane (above) and its downstream cross-sectional plane (below) for subject 1: (a1, a2) standard k-*ε* solution; (b1, b2) standard k-*ω* solution; (c1, c2) k-*ω* SST solution; (d1, d2) LES solution.

**Figure 6:** Axial velocity distribution (m/s) in the minimum cross-sectional plane (above) and its downstream cross-sectional plane (below) for subject 2: (a1, a2) standard k-*ε* solution; (b1, b2) standard k-*ω* solution; (c1, c2) k-*ω* SST solution; (d1, d2) LES solution.

**Figure 7:** The LES and unsteady RANS comparisons of the mean static pressure distribution corresponding to its cross-sectional area from the nasopharynx to epiglottis for subject 1: (a) before surgery and (b) after surgery.

**Figure 8:** The LES and unsteady RANS comparisons of the mean static pressure distribution corresponding to its cross-sectional area from the nasopharynx to epiglottis for subject 2: (a) before surgery and (b) after surgery.

**Figure 9:** The LES and unsteady RANS comparisons of wall shear stress in a point located on the anterior side downstream of the minimum cross-sectional area: (a) subject 1 before surgery and (b) subject 1 after surgery.

**Figure 10:** The LES and unsteady RANS comparisons of wall shear stress in a point located on the anterior side downstream of the minimum cross-sectional area: (a) subject 2 before surgery and (b) subject 2 after surgery.

**Figure 11:** Comparison of wall shear stress time series at the larynx for two OSA subjects: (a) subject 1 and (b) subject 2.

**Figure 12:** Spectral analysis of wall shear stress time series at the larynx for two OSA subjects with frequency from 2.5 Hz to 6 Hz: (a) subject 1 and (b) subject 2.

**Table 1:** Severity indices of OSA.

	AHI (events/h)	O_2_ saturation (%)
Normal	<5	>95
Mild	5-19	>85
Moderate	20-39	>65
Severe	>40	<65

**Table 2:** AHI measurement, minimal cross-sectional area near the retropalate, maximal cross-sectional area in the oropharynx, and area ratio (AR) (min area/max area) of two OSA subjects.

Subject	State	AHI	Min area (mm^2^)	Max area (mm^2^)	Area ratio
Subject 1	Presurgery	64.8	53	256.4	0.21
	Postsurgery	15.8	100	264.1	0.38

Subject 2	Presurgery	60.7	46	241.8	0.19
	Postsurgery	23.9	318	645.0	0.49

## Data Availability

This work was carried out in strict accordance with the recommendations of the National Institutes of Health, and the protocol was approved by the Tongren Hospital of the Capital Medical University.
